The article "Analysis of the Curative Effect and Influencing Factors of Collagen Sponge Combined with Autologous Skin Graft in the Treatment of Deep Burn Patients" was retracted in 2023. Reasons: signs of a paper mill; suspected computer-generated content; unreliable results or conclusions; concerns about the data.

# Analysis of the Curative Effect and Influencing Factors of Collagen Sponge Combined with Autologous Skin Graft in the Treatment of Deep Burn Patients

**DOI:** 10.1155/2021/6963401

**Published:** 2021-10-26

**Authors:** Jian Cai, Duyin Jiang, Wei Zang

**Affiliations:** Department of Emergency, The Second Hospital of Shandong University, Jinan, Shandong 250033, China

## Abstract

Burn is one of the common traumatic diseases in clinics. After deep burn, the complicated changes of the condition are caused by the burn wound, which ends with the repair of the wound. For patients with deep burns, whether the wound can be repaired as soon as possible is the key to the success of clinical treatment. For patients with deep burns, due to the lack of an autologous skin source, scar hyperplasia at donor site, skin graft repair at donor site, postoperative flap necrosis, and other problems in traditional surgical procedures, the method of improving function only by an autologous skin source has been unable to perform the later function reconstruction in patients with deep burns. In this study, collagen sponge combined with autologous skin graft was used to treat patients with deep burn, and the clinical efficacy of the patients was observed, and the related factors affecting the efficacy of the patients were analyzed. The results showed that collagen sponge combined with autologous skin graft was effective in the treatment of deep burn patients, and it was worth popularizing. Deep III-IV degree burns, wound infection, and hospital stay >3 months are all risk factors affecting the postoperative curative effect of patients. Therefore, in the clinical work, we should focus on patients with deep III-IV degree burns, perform surgery as soon as possible, and actively deal with wounds to prevent infection, which is beneficial to improve the curative effect.

## 1. Introduction

Burn mainly refers to the damage of the skin and mucous membrane caused by high temperature, electric current, and radiation. It is one of the most common traumatic diseases in clinics, which can cause great changes in the pathophysiology of patients, and its disability rate and mortality rate are high. It has become one of the major public health problems in the world [1, 2]. Clinically, the main cause of death of burn patients is often the infection caused by a large number of necrotic tissues attached to the wound surface. Early surgical methods are used to remove the dead burn necrotic tissues, that is, escharectomy, combined with skin grafting to seal the open wound surface [3, 4]. With the improvement of people's living standards and the progress of science and technology, the treatment of burn patients is not limited to saving lives. How to repair the wounds faster and with higher quality, let the patients return to society, and improve their functions and physical appearance after healing are the ultimate goals of treatment [5, 6]. Deep burns refer to burns that need more than 21 days for the wound to heal itself, including deep second-degree burns, third degree burns, and fourth degree burns. Skin grafting is the main treatment. Deep burn often requires multiple debridement and skin grafting to repair the wound, and scar hyperplasia and contracture often accompany the wound healing, which seriously affects the patient's quality of life. At present, the main method to solve the dysfunction caused by scar contracture is skin graft after scar resection, while patients with deep burns are often faced with the problem of severe shortage of their own skin sources [7, 8]. In recent years, with the development of tissue engineering, medical collagen sponge has been widely used in the field of wound repair. Collagen, as a natural polymer, is abundant in various tissues of human body including the skin, blood vessels, tendons, cartilages, and bones. Collagen is not only abundant in human body but also plays an important role in maintaining normal cell function, skin elasticity, muscle strength and toughness, and tissue repair [9, 10]. The purpose of this study is to investigate the efficacy of collagen sponge combined with autologous skin graft in the treatment of patients with deep burn and to analyze the related factors affecting the efficacy. Specific reports are as follows.

The article "Analysis of the Curative Effect and Influencing Factors of Collagen Sponge Combined with Autologous Skin Graft in the Treatment of Deep Burn Patients" was retracted in 2023. Reasons: signs of a paper mill; suspected computer-generated content; unreliable results or conclusions; concerns about the data.

## 2. Materials and Methods

### 2.1. Patients

284 patients with deep burn admitted to our hospital from June 2016 to February 2021 were selected as research objects. Among them, there were 166 males and 118 females with an average age of (43.54–16.75) years, ranging from 18 to 69 years. The total burned area was 36.53–84.68% total body surface area (TBSA), and the average burned area was (60.08 ± 19.48) % TBSA. The third degree burn area was 14.54–53.85% TBSA, and the average III degree burn area was (33.56 ± 9.51) % TBSA. Causes of burns: 74 cases of flame burns, 96 cases of hydrothermal burns, 42 cases of chemical burns, and 72 other cases. Burn sites: 124 arms and legs, 68 trunks, and 92 head and face. Inclusion criteria: total burn area ≥30% TBSA, and III degree burn area ≥10% TBSA, those who have not received surgery in the outer hospital, hospitalized within 24 hours after burn, and complete clinical data. Exclusion criteria: those with diabetes and other basic diseases; complicated with abnormal heart, liver, and kidney functions, pregnant and lactating women, those with hematological diseases, follow-up of patients with process loss.

The article "Analysis of the Curative Effect and Influencing Factors of Collagen Sponge Combined with Autologous Skin Graft in the Treatment of Deep Burn Patients" was retracted in 2023. Reasons: signs of a paper mill; suspected computer-generated content; unreliable results or conclusions; concerns about the data.

### 2.2. Treatment Methods

All patients were treated with collagen sponge combined with autologous skin graft. After admission, the scab, necrotic tissue, and attached infectious substances were removed from the wound surface in the dressing room, the chlorhexidine solution was washed and disinfected, and the blisters were drained. According to the condition of the wound surface, the sterile medical gauze soaked with sulfadiazine silver cream or compound polymyxin B ointment and purple grass oil was used to bind the wound surface. The patients were rehydrated according to Ruijin formula to resist shock, the standby body was out of shock, the water and electrolyte were stable, the wound surface was not seriously infected, and the operation was performed in the operating room when the limit of subcutaneous edema was clear. Cut the corresponding area of medical collagen sponge to cover the wound. All the cases in this study were treated with continuous closed negative pressure drainage (VSD). The VSD device covered the wound surface, and the tightness was intact. Set the negative pressure to 10–15 kPa, slowly drip 0.9% sodium chloride solution or low-concentration skin disinfectant solution from the lavage end of the self-pressure device to wash the wound surface, 500–1000 mL per day, and the wound surface is continuously attracted by negative pressure. Routine anti-infection treatment was given after debridement. After early debridement and VSD treatment, the VSD device was replaced once every 6–8 days. While replacing the VSD device, remove undegraded medical collagen sponge, keep granulation tissue, and continue to cover the wound with medical collagen sponge (Wuxi Brady Biological Engineering Co., Ltd.). After the wound surface is covered with fresh granulation tissue, scrape or cut the granulation tissue higher than the skin around the wound, without completely scraping the granulation, slightly trim the periphery of the wound to form a steep edge, so as to prevent the skin graft edge from protruding from the wound edge. Disinfect the wound with iodophor, rinse it with 0.9% sodium chloride solution, and apply it wet for later use. According to the size of the wound, the thick skin of the body blade was cut out and punctured appropriately for later use. Flatten and apply the prepared skin patch to the wound surface with proper tension and sew and fix the skin patch with a skin nailing machine or silk thread. 0.9% sodium chloride solution was used to wash the subcutaneous wound, and Vaseline gauze was used to cover the skin. After that, the VSD device was installed and the film was sealed.

The article "Analysis of the Curative Effect and Influencing Factors of Collagen Sponge Combined with Autologous Skin Graft in the Treatment of Deep Burn Patients" was retracted in 2023. Reasons: signs of a paper mill; suspected computer-generated content; unreliable results or conclusions; concerns about the data.

Routine anti-infection treatment with sensitive antibiotics was given after operation, and the negative pressure was set at 10–15 kPa. Dismantle the VSD device in 6–8 days. The residual wound was covered with Vaseline gauze and pressurized with elastic bandage, and the dressing was changed once every 2-3 days until the residual wound healed.

### 2.3. Observation Indicators

All patients were followed up for more than 6 months after operation, and the curative effect was evaluated. According to the healing condition of skin graft, the curative effect was evaluated: excellent: the skin color of wound margin and skin graft was normal, the scar width was less than <0.5 cm, the functional activity was good, and people could take care of themselves in daily life; good: the skin color of wound margin and skin is close to normal, the scar width is 0.5–1 cm, and it is difficult to take care of yourself in daily life; fair: the skin color of the wound margin and skin is abnormal, the scar width is 1.0–2.0 cm, and daily life cannot take care of itself; poor: scar hyperplasia was obvious on the wound surface, and the scar width was >2.0 cm. Excellent and good rate = (excellent + good) cases/total cases × 100%.

According to the curative effect, all patients were divided into the excellent and good group (*n* = 258) and fair and poor group (*n* = 26). The clinical data such as gender, age, educational level, marital status, burn cause, burn location, burn degree, wound infection, and hospital stay were recorded. The related factors affecting the curative effect of patients were analyzed by univariate analysis and multivariate analysis.

### 2.4. Statistical Methods

The results of this experiment were statistically analyzed by SPSS 20.0 (SPSS Co., Ltd., Chicago, USA). Count data were expressed by (rate), and the chi-square test was used for their comparison between groups. Measurement data were expressed by (mean ± standard deviation), and the *t*-test was used for their comparison between groups. Multivariate analysis adopts the multiple logistic regression model. *P* < 0.05 indicates that the difference is statistically significant.

## 3. Results

### 3.1. Postoperative Efficacy of Patients

The wound healing time of all patients was (25.74 ± 5.92) d, and the hospital stay was (2.46 ± 0.95) months. 6 months after operation, among 284 patients, 98 were excellent, 160 were good, 22 were fair, and 4 were poor, and the excellent and good rate was 90.85% (258/284), as given in Table 1.

### 3.2. Typical Cases

Typical case 1: A 33-year-old man presented with a hot press injury to his left upper limb. The wounds were covered with VSD after thorough debridement. After 10 days, the dressing was opened, and the wound granulation tissue grew satisfactorily. Twelve days later, a flap transfer combined with free skin grafting was performed, as shown in Figure 1. Typical case 2: A 1-year-old and 6-month-old man presented with a hydrothermal burn on his right lower limb. After thorough debridement and hemostasis, the wound was covered with VSD. After 7 days, the wound granulation tissue grew well. After 10 days, the free skin graft was used for repair and the wound was closed, as shown in Figure 2.

The article "Analysis of the Curative Effect and Influencing Factors of Collagen Sponge Combined with Autologous Skin Graft in the Treatment of Deep Burn Patients" was retracted in 2023. Reasons: signs of a paper mill; suspected computer-generated content; unreliable results or conclusions; concerns about the data.

### 3.3. Univariate Analysis of Influencing the Postoperative Curative Effect of Patients

Univariate analysis showed that age, burn degree, wound infection, and hospital stay were all related to the postoperative curative effect (*P* < 0.05), as given in Table 2.

### 3.4. Multivariate Analysis of Influencing the Postoperative Curative Effect of Patients

Multivariate logistic analysis showed that deep III-IV degree burns, wound infection, and hospital stay >3 months were all risk factors affecting the postoperative curative effect (*P* < 0.05), as given in Tables 3-4.

## 4. Discussion

Burn is one of the common traumatic diseases in clinics. After deep burn, the complicated changes of the condition are caused by the burn wound, which ends with the repair of the wound. For patients with deep burns, whether the wound can be repaired as soon as possible is the key to the success of clinical treatment [11, 12]. In order to improve the cure rate, one of the key measures is to cut and implant the skin at an early stage and close the plane as soon as possible. For many years, the key to improving the treatment level of deep burn is to clear the wound surface in time, close the wound surface as soon as possible, prevent shock and infection, and reduce complications. However, in the later stage, the burned site and skin graft area of the patient will appear as obvious scar hyperplasia, functional site contracture deformity, local repeated tension blisters, and repeated scar rupture to form chronic ulcer. Patients lose the most basic living ability such as toilet, eating, and walking, which bring many problems to rehabilitation exercise and functional reconstruction treatment and seriously affect the quality of life of patients [13, 14]. Traditional surgical methods for treating scar contracture after deep burn are as follows: (1) transfer skin flap to directly transfer soft scar tissue or normal skin tissue around. Although it can repair a large skin defect, the donor area damaged greatly, so it is possible to repair it by skin grafting. After healing, obvious scars will be left behind, resulting in the inability to provide the skin again, and the appearance and shape after operation are bloated, so it is necessary to perform skin flap repair in the later stage. (2) Scar reconstruction: Z-shaped plastic surgery is commonly used. However, the effect of scar reconstruction in relieving scar contracture is limited, and the probability of necrosis of skin flap is very high. (3) The expanded scar flap is to select the soft scar skin around the operation area for primary dilator implantation, and after the wound heals, it will be expanded to an ideal state at regular intervals and then undergo secondary operation. After the scar in the functional part is released, the expanded scar flap will be used to repair the wound. Because of the full-thickness structure of the expanded skin flap, the function and beauty of the transplanted site can be improved obviously. However, the production cycle of the expanded scar skin is longer (3–6 months), which may lead to ischemia and necrosis of the scar skin during expansion, and the embedded dilator may also be broken, infected, and displaced, thus causing great damage to the donor skin area [15, 16]. Therefore, for patients with deep burn, because of the shortage of autologous skin source, scar hyperplasia in donor area, skin graft repair in donor area, and skin flap necrosis after operation, the method of improving the function of patients with deep burn only by an autologous skin source can no longer be competent for the later functional reconstruction.

The article "Analysis of the Curative Effect and Influencing Factors of Collagen Sponge Combined with Autologous Skin Graft in the Treatment of Deep Burn Patients" was retracted in 2023. Reasons: signs of a paper mill; suspected computer-generated content; unreliable results or conclusions; concerns about the data.

The basic process of wound healing includes cell proliferation, extracellular matrix reconstruction, and inflammatory reaction, which all need to conform to the microenvironment of cell growth. Any factors affecting these processes and environment will affect wound healing. The local microenvironment includes certain temperature, humidity, pH, and various nutrients. Preventing local infection is also one of the important conditions to ensure tissue repair. How to accelerate wound healing, relieve pain, and reduce scar formation is of great significance to improve the quality of wound healing [17, 18]. Therefore, wound coverage is one of the most important issues in wound treatment. The ideal covering material should have the following characteristics: strong adhesion, promoting wound healing, and resisting infection [19, 20]. With the development of bioengineering and materials science, the application of biomaterials has brought new breakthroughs in wound repair and functional reduction technology [21, 22]. Collagen sponge, as a natural biomaterial, is nontoxic, and its degradation products can be absorbed by the body without causing harm to the body. Collagen sponge has a morphological structure similar to dermis and has good water permeability and air permeability. Low antigenicity and good biocompatibility can be used for wound coverage for a long time. It has a reticular porous structure, which paves the way for the migration and proliferation of epidermal cells on the wound surface, is beneficial to the proliferation and repair of cells, and accelerates the healing of the wound surface. Collagen sponge is a growth-promoting factor of fibroblasts and vascular endothelial cells. It can promote capillary formation, accelerate granulation tissue growth, and provide abundant nutrients for tissue growth [23, 24].

The article "Analysis of the Curative Effect and Influencing Factors of Collagen Sponge Combined with Autologous Skin Graft in the Treatment of Deep Burn Patients" was retracted in 2023. Reasons: signs of a paper mill; suspected computer-generated content; unreliable results or conclusions; concerns about the data.

The results of this study showed that among the 284 patients, 98 were excellent, 160 were good, 22 were fair, and 4 were poor, and the excellent and good rate was 90.85% (258/284). It shows that collagen sponge combined with autologous skin graft is effective in treating deep burn patients. The reasons are as follows: collagen sponge is beneficial to promote the growth of wound granulation tissue; collagen sponge adsorbs the active tissue cells in wound exudate to the wound base, while inactivated tissue cells are fully drained by the VSD device, so as to prevent necrosis and aggregation of infected tissues, keep the wound clean, reduce antibiotic dosage, improve local microenvironment, and promote the growth of granulation tissue. Collagen sponge is also beneficial to promote wound hemostasis, and it can be tightly adhered to the wound and mechanically seal the capillary opening. At the same time, collagen molecules adsorb and aggregate platelets, activate coagulation factors, start the endogenous hemostasis pathway, and promote postoperative wound hemostasis. Moreover, collagen sponge only produces hemostasis locally, does not activate the whole body coagulation system, does not increase the risk of deep vein thrombosis, and is relatively safe. Collagen sponge can also be degraded and absorbed. The final degradation products of collagen are essential amino acids, which can be absorbed by the body and provide nutrition for tissue growth and wound repair. Therefore, the application of collagen sponge is beneficial to accelerate the healing of patients' wounds.

The univariate analysis showed that age, burn degree, wound infection, and hospital stay were all related to the postoperative curative effect. Multivariate logistic analysis showed that deep III-IV degree burn, wound infection, and hospital stay >3 months were all risk factors affecting the postoperative curative effect. The reason is that the more serious the burn, the more serious the body injury and the weaker the body's self-repair ability, which leads to a poor skin recovery effect and affects the curative effect [25]. Therefore, the patients with III-IV degree burn should be treated as early as possible to reduce complications and improve clinical efficacy. The necrotic tissue of burn wound provides a good culture medium for bacteria. It is the main source of wound infection, and the damage of immune function after burn also returns to normal after wound healing or escharectomy and skin grafting. Therefore, active treatment of wounds (including escharectomy, skin grafting, and topical drugs to promote wound healing) is the key to prevent infection. Because of the need to recover from bed after burns, skin grafts often use lower extremity skin grafts, and extensive dressings after surgery restrict the patient's movement, which greatly increases the risk of deep vein thrombosis in the lower extremities, thereby affecting the efficacy.

The article "Analysis of the Curative Effect and Influencing Factors of Collagen Sponge Combined with Autologous Skin Graft in the Treatment of Deep Burn Patients" was retracted in 2023. Reasons: signs of a paper mill; suspected computer-generated content; unreliable results or conclusions; concerns about the data.

## 5. Conclusion

Collagen sponge combined with autologous skin graft is effective in treating patients with deep burn, which is worth popularizing. Deep III-IV degree burns, wound infection, and hospital stay >3 months are all risk factors affecting the postoperative curative effect of patients. Therefore, in the clinical work, we should focus on patients with deep III-IV degree burns, perform surgery as soon as possible, and actively deal with wounds to prevent infection, which is beneficial to improve the curative effect.

## Figures and Tables

**Figure 1:** Typical case 1. (a) The wound surface after debridement of the left upper limb heat compression injury. (b) The wound covered by VSD. (c) The wound granulation tissue grew satisfactorily after the 10^th^ day of VSD coverage. (d) The wound surface observed 1 month after skin graft transplantation.

**Figure 2:** Typical case 2. (a) The wound surface after debridement of the right lower extremity heat burn. (b) The wound covered by VSD. (c) After 1 week of VSD, the granulation tissue grew satisfactorily. (d) After skin graft for 3 months, skin graft survived well.

**Table 1:** Postoperative efficacy of patients.

Patients	Excellent	Good	Fair	Poor	Excellent and good rate
*n*	98	160	22	4	90.85% (258/284)

**Table 2:** Univariate analysis of influencing the postoperative curative effect of patients.

Factors	*n*	Excellent group (*n* = 258)	Poor group (*n* = 26)	*t*/*χ*^2^	*P*
Gender				1.369	0.242
Male	166	148 (57.36)	18 (69.23)		
Female	118	110 (42.64)	8 (30.77)		
Age (years)	284	42.82 ± 17.04	50.68 ± 16.82	2.244	0.026
Degree of education				0.675	0.411
High school and above	195	179 (69.38)	16 (61.54)		
Junior high school and below	89	79 (30.62)	10 (38.46)		
Marital status				0.128	0.938
Unmarried	58	52 (20.16)	6 (23.08)		
Married	182	166 (64.34)	16 (61.54)		
Widowed/divorced	44	40 (15.50)	4 (15.38)		
Causes of burns				0.514	0.916
Flame	74	68 (26.36)	6 (23.08)		
Hydrothermal	96	88 (34.11)	8 (30.77)		
Chemistry	42	38 (14.73)	4 (15.38)		
Others	72	64 (24.80)	8 (30.77)		
Burn site				0.142	0.932
Arms and legs	124	113 (43.80)	11 (42.31)		
Trunk	68	61 (23.64)	7 (26.92)		
Head and face	92	84 (32.56)	8 (30.77)		
Degree of burn				5.724	0.017
Deep II degree	105	101 (39.15)	4 (15.38)		
Deep III-IV degree	179	157 (60.85)	22 (84.62)		
Wound infection				13.153	<0.001
Yes	48	37 (14.34)	11 (42.31)		
No	236	221 (85.66)	15 (57.69)		
Hospital stay (months)				6.476	0.039
<1	96	90 (34.88)	6 (23.08)		
1–3	124	115 (44.58)	9 (34.61)		
>3	64	53 (20.54)	11 (42.31)		

The article "Analysis of the Curative Effect and Influencing Factors of Collagen Sponge Combined with Autologous Skin Graft in the Treatment of Deep Burn Patients" was retracted in 2023. Reasons: signs of a paper mill; suspected computer-generated content; unreliable results or conclusions; concerns about the data.

**Table 3:** Assignment for multivariate analysis of factors.

Factors	Variable	Assignment
Age	X1	Continuous variable
Degree of burn	X2	Deep II degree = 0, deep III-IV degree = 1
Wound infection	X3	No = 0, yes = 1
Hospital stay	X4	<1 = 0, 1–3 = 1, >3 = 2

**Table 4:** Multivariate analysis of influencing the postoperative curative effect of patients.

Variables	B	S.E	Wald	*P*	OR	95% CI
Age	0.436	0.198	2.086	0.203	1.547	0.974–1.921
Degree of burn	1.056	0.582	5.137	0.024	2.875	1.633–3.985
Wound infection	1.368	0.346	6.325	0.016	3.927	1.964–6.082
Hospital stay	0.935	0.492	4.398	0.045	2.547	1.358–3.416

## Data Availability

The data used to support the findings of this study are available from the author upon request.
